The article "Network Pharmacology-Based Analysis on Lonicera japonica for Chronic Osteomyelitis Treatment" was retracted in 2023. Reasons: unreliable results or conclusions; concerns about the data; concerns about the peer review; concerns about the citations.

# Network Pharmacology-Based Analysis on *Lonicera japonica* for Chronic Osteomyelitis Treatment

**DOI:** 10.1155/2022/1706716

**Published:** 2022-01-24

**Authors:** Tingting Shao, Kai Huang

**Affiliations:** ^1^Infectious Disease Department, Tongde Hospital of Zhejiang Province, 234# Gu-cui Road, Hangzhou 310012, China; ^2^Department of Orthopedics, Tongde Hospital of Zhejiang Province, 234# Gu-cui Road, Hangzhou 310012, China

## Abstract

**Materials and Methods:**

Active compounds of LJP were examined established on the analysis platform, Traditional Chinese Medicine Systems Pharmacology (TCMSP) database. DrugBank identified drug targets and annotated them on UniPort and GeneCards. Besides, the COM-related genes were identified on GeneCards. The network of the drug, main active compounds, targets, and diseases was built utilizing Cytoscape. STRING was utilized to build the protein-protein interaction network. Moreover, the KEGG and GO pathway enrichment analysis were applied to analyze biological function.

**Results:**

23 active compounds of LJP were screened, and 204 drug targets and 686 COM-related genes were identified. Forty-five intersection genes were overlapped from 204 drug targets and 686 COM-related genes. The drug-active compounds-target protein-diseases network was established based on 23 active compounds of LJP and 45 intersection genes. Moreover, the interaction of 45 intersection genes was explored by the PPI network, and the drug-active compounds-target protein-diseases network was formed grounded by 23 active compounds of LJP, 45 intersection genes, and PPI network. The KEGG and GO pathway enrichment analysis specified that 45 intersection genes primarily enriched in immune-related pathways and oxidative stress-related pathways.

**Conclusions:**

In the research done, the main active compounds of LJP and drug targets in the treatment of COM were identified. Our findings might provide the ingredient option of LJP and drug targets of LJP in COM treatment.

## 1. Introduction

Chronic osteomyelitis (COM) is an autoinflammatory condition which characteristics as osseous infection and with or without neighboring soft tissues infection [1]. It is difficult to treat and has high morbidity and mortality due to its stubbornness [2]. The main reason for COM included trauma and postoperative infection, so it exhibited continuous focus invasion, hematogenous spread, and vascular insufficiency after infecting microorganisms [3]. COM usually persists intermittently for months or years, with multiple clinical failures and relapses after periods of quiescence and apparently successful treatment [4]. The prolonged inflammatory process not only increases the risk of malignant transformation but also increases the risk of suicide of COM patients, having a big effect on patients' life quality and healthcare system costs [3]. Nowadays, the treatment of chronic osteomyelitis mainly includes systemic treatment and local treatment, such as systemic antibiotics, bacterial immunotherapy, debridement surgery, and so on. However, the use of antibiotics may lead to serious side effects, and surgery does not guarantee that the infection will be completely cleared. The treatment of COM remains a difficult and challenging problem for orthopaedic surgeons and infectious diseases specialists.

The article "Network Pharmacology-Based Analysis on Lonicera japonica for Chronic Osteomyelitis Treatment" was retracted in 2023. Reasons: unreliable results or conclusions; concerns about the data; concerns about the peer review; concerns about the citations.

In recent years, traditional Chinese medicines (TCMs) show obvious therapeutic effects and advantages in many disease treatments [5, 6]. For instance, andrographolide alleviates oxidative stress and inflammation in arthritis [7], flavonoids promote bone repair in COM [8], and betulinic acid relieves synovial inflammation in arthritis [9]. *Lonicera japonica* (LJP) is a TCM that is widely used for the treatment of fever, carbuncle, and tumors, and so on; including COM, it significantly exhibits functions of antioxidation, antibacteria, anti-inflammation, and immunoregulation [7, 10, 11]. However, like other TCM, LJP possesses a synergistic effect and multipathway, multitarget, and multicomponent characteristics that produce indistinct mechanisms of action, uncertain substance bases, and other problems, which result in unclear molecular mechanisms for treating COM. So, it is significant to investigate LJP drug targets and active compounds which will be a great help for COM efficient precise treatment and drug selection.

Network pharmacology is a combined multidisciplinary idea investigating synergistic impacts and potential methods of various mixtures via evaluating complicated and multilayered networks, that is a pharmacology and pharmacodynamics-based novel research field [12]. In the research conducted, we established a thorough network pharmacology attempt to investigate the possible LJP pharmacological mechanism on COM by network evaluation and molecular docking. LJP active compounds were examined, and target proteins were anticipated and assessed. The COM-related genes were screened in the meantime. After that, the protein-protein interaction (PPI) and drug-compounds-genes-disease network were built to cross-validate the target proteins, and the Kyoto Encyclopedia of Genes and Genomes (KEGG) pathway and analyses and gene ontology (GO) were established for target proteins. We intended to discover potential key targets of LJP for COM treatment.

## 2. Materials and Methods

### 2.1. Screening Bioactive Components in LJP

LJP active components were examined from the Traditional Chinese Medicine Systems Pharmacology Database and Analysis Platform (TCMSP, https://tcmspw.com/index.php) [13]; furthermore, antiosteomyelitis components [14] identification was done with the ADME parameter-based virtual screening of components. In a previous study, molecules with oral bioavailability (OB) ≥ 30% were believed as a good OB, and a drug likeness of (DL) ≥ 0.18 [15] was to define active molecules. LJP active components were assessed established on the cutoff value as OB ≥ 30% and DL ≥ 0.18 in our study.

The article "Network Pharmacology-Based Analysis on Lonicera japonica for Chronic Osteomyelitis Treatment" was retracted in 2023. Reasons: unreliable results or conclusions; concerns about the data; concerns about the peer review; concerns about the citations.

### 2.2. Screening LJP Active Compound Targets

LJP active compound targets were screened in DrugBank [16], and the targets were annotated by UniPort [17] and GeneCards databases [18].

### 2.3. Screening of COM-Related Genes

The COM-related genes were screened by GeneCards databases (https://www.GeneCards.org) through querying with keywords chronic osteomyelitis and COM.

### 2.4. Construction of the Drug-Compounds-Genes-Disease Network

The intersection genes between LJP active compound targets and COM-related genes were overlapped. Then, the interaction network of the drug, compounds, genes, and disease was constructed and visualized using Cytoscape3.8.0 [19]. Edge and node comprised this network. Molecules are represented as nodes (diseases, signal pathways, protein targets, or compounds), and intermolecular interactions are characterized as edges (diseases, signal pathways, protein targets, or compounds), namely, the connections between nodes.

### 2.5. PPI Network Construction

Online STRING 11.0 (https://string-db.org/) was incorporated to analyze COM-related target proteins for PPI network construction. Protein-protein interactions with confidence score ranges were predicted from the STRING database (low confidence score <0.4; medium: 0.4–0.7; high >0.7–0.9; highest confidence >0.9) [20].

### 2.6. GO and KEGG Pathway Analysis

KEGG pathway analysis and GO function were completed using cluster Profiler R package 3.8.1 with FDR <0.2 and *P* value <0.05 (FDR, false discovery rate) [21]. GO annotation contains the biological process (BP), molecular functions (MF), and cellular components (CC).

## 3. Results

### 3.1. LJP Active Compounds and Predicted Targets

The TCMSP database (satisfied the criteria of OB ≥ 30% and DL ≥ 0.18) was applied for the identification of twenty-three active compounds of LJP (Table 1). Among the 23 active compounds of LJP, we found 204 target proteins (Supplementary Table 1), such as chryseriol included NOS2, PTGS2, and MAPK14 (Table 2). The target proteins of active compound luteolin included PTGS2, EGFR, AKT1, VEGFA, MMP9, IL-10, and IL-6 (Table 2). These outcomes indicated the LJP primary active compounds generally regulated immune-related genes.

The article "Network Pharmacology-Based Analysis on Lonicera japonica for Chronic Osteomyelitis Treatment" was retracted in 2023. Reasons: unreliable results or conclusions; concerns about the data; concerns about the peer review; concerns about the citations.

### 3.2. Identification of COM-Related Genes

We also identified 686 COM-related genes from the GeneCards database, the score ranges from 0.44 to 78.550, the median value is 7.945, and the mean value is 11.065 (Supplementary Table 2). The top 10 COM-related genes included TNF, IL-1RN, IL-6, IL-1*β*, IL-10, IFNG, NLRP3, CYBB, TERT, and TNFSF11 (Table 3).

### 3.3. Building of the Drug-Active Compounds-Target Protein-Diseases Network

According to the previous analysis, there were 45 intersection genes overlapped between 686 target proteins of LJP active compound and 204 COM-related genes (Figure 1(a)). The overlapped genes included immune-related genes (VEGFA, MMP9, IL-10, IL-6, and MMP1), chemokines (CCL2, CXCL2, CXCL8, and CXCL10), and other genes. Then, the drug-active compounds-target protein-diseases network was established based on 15 main active compounds of LJP and 45 overlapped genes between target proteins and COM-related genes (Figure 1(b)). We found that chryseriol, luteolin, quercetin, kaempferol, beta-carotene, and beta-sitosterol were the primary COM treatment active components.

### 3.4. Identification of the Hub Genes in the Drug-Active Compounds-Target Protein-Diseases Network

Furthermore, investigate the interaction of 45 overlapped genes by building a PPI network. It was discovered that the network included 45 nodes and 557 edges with an interaction score >0.4 (Figure 2(a)). 45 nodes represented the intersection genes between target proteins of active compound of LJP and COM-related genes, and 557 edges represented interaction relationship. We found that ALB, AKT1, IL-6, VEGF, MMP9, and CCL2 showed a high connection degree (Figure 2(b)).

### 3.5. GO Function and KEGG Enrichment Examination of the Target Proteins

The overlapped genes mechanism was further explored by KEGG pathway enrichment and GO function evaluation. We found that the upregulated overlapped genes primarily enriched in immune-related processes and oxidation-reduction processes, such as leukocyte migration, T cell activation, and reply to reactive oxygen species. Cellular components included membrane microdomain, membrane raft, and so on. Molecular functions included antioxidant activity, receptor-ligand activity, and cytokine receptor binding (Figure 3(a)). According to KEGG pathway evaluation, the top 10 pathways are primarily supplemented in immune-related pathways, including the IL-17 signaling pathway, fluid shear stress, and atherosclerosis, AGE-RAGE signaling pathway in diabetic complications (Figure 3(b)).

## 4. Discussion

COM is an inflammatory disorder of the bone marrow with progression tendencies, including the often periosteal tissues and cortical plates [22]. In the majority of cases, a combined medical and surgical approach is required for chronic osteomyelitis treatment [4]. The medical approach usually needs a long course of targeted antibiotic therapy. However, due to high failure and recurrence rates, new treatments and drugs are needed to be found for COM.

The article "Network Pharmacology-Based Analysis on Lonicera japonica for Chronic Osteomyelitis Treatment" was retracted in 2023. Reasons: unreliable results or conclusions; concerns about the data; concerns about the peer review; concerns about the citations.

Currently, broad use of TCM has revealed obvious therapeutic effects and advantages in inflammatory bone diseases treatment, including osteoarthritis [23], rheumatoid arthritis [24], and COM [25]. In our previous study, we combined wuweixiaodu drink with surgery and antibiotics administration for the patients with traumatic chronic tibial osteomyelitis and discovered that wuweixiaodu drink could mitigate traumatic CO local lesions with general status amelioration, resulting in significant effectiveness [26]. What is more, as an important TCM in wuweixiaodu drink, LJP and its active principles have been confirmed to hold broad pharmacological actions, including activities such as antioxidative, antibacterial, antiviral, and anti-inflammatory [27]. These activities have a vital part in the COM treatment. Though, LJP underlying the molecular mechanism, drug targets, and active compounds are still uncertain.

In the present research, we identified a total of 23 active compounds of LJP including chryseriol, luteolin, eriodyctiol, kaempferol, beta-carotene, quercetin, and so on. In addition, 204 targets of LJP and 608 COM-related genes were predicted and identified. Then, 45 interaction genes between targets of LJP and COM-related genes were overlapped, including immune-related genes (VEGFA, MMP9, IL-10, IL-6, and MMP1), chemokines (CCL2, CXCL2, CXCL8, and CXCL10), and other genes. We further constructed the network of drugs, compounds, targets, and diseases. The network indicated that beta-sitosterol, beta-carotene, luteolin, kaempferol, and quercetin were the primary active compounds of LJP in COM treatment. Moreover, the PPI network of 45 intersection genes was constructed. ALB, AKT1, IL-6, VEGFA, MMP9, CCL2, IL-1*β*, PTGS2, CXCL8, and ICAM1 were identified as the hub genes. Furthermore, to analyze the mechanism of LJP in COM treatment, it was discovered that hub genes were primarily supplemented in immune-related and pathways and oxidative stress-related pathways.

According to our result, luteolin is a main activate compound from LJP, and its target proteins include IL-6, IL-10, MMP9, VEGFA, AKT1, EGFR, and so on. IL-10 mostly bears immune regulatory functions. Sigrun et al. reported that reducing the expression of IL-10 contributes to enhanced subsequent-1*β* release and inflammasome activation [28]. IL-1*β* and IL-6 are the main COM-related genes identified in our study. As important proinflammatory cytokines, IL-1*β* and IL-6 directly participate in osteoclast activity regulation and bone desorption that happen in osteomyelitis and could consequently be a vital part of its pathogenesis [29]. So, we could hypothesize that a therapeutic effect on COM may be played by luteolin, through regulating the level of IL-10, IL-6, and IL-1*β*. In the study of Soung, postoperative exudates of chronic suppurative osteomyelitis demonstrated constantly enhanced angiogenesis-related proteins expression, including VEGFA [30], which is another target protein of luteolin. It was indicated that wound healing signaling was activated via increased activation angiogenesis [30]. It was already known that angiogenesis increased in various chronic infection mouse models [31], and a considerable rise in high-grade infection incidences during osteomyelitis formation was reduced gradually by boosting angiogenesis and humoral immunity. So, luteolin may promote wound healing through increasing angiogenesis by regulating VEGFA. As an infectious bone disease, COM is a dysregulation of bone formation and resorption, which results in excessive bone resorption. Akt signaling is critical for osteoclast differentiation and apoptosis, which is a vital part of osteomyelitis [32, 33]. MMP9 is an osteoclast-specific gene and involves in the degradation of the bone matrix during bone resorption [34]. It has been proved that EGFR signaling is vital for differentiation, proliferation, and survival of osteoblastic cells [35]. Ji et al. reported that EGFR signaling can mediate *Staphylococcus aureus* (*S. aureus*) internalization by osteoblasts [36], which is a vital part of osteomyelitis recurrence and persistence. So, Akt, MMP9, and EGFR play a vital part in COM pathogenesis through bone resorption regulation. Luteolin may prevent bone resorption by regulating the level of Akt, MMP9, and EGFR, so as to treat COM.

The article "Network Pharmacology-Based Analysis on Lonicera japonica for Chronic Osteomyelitis Treatment" was retracted in 2023. Reasons: unreliable results or conclusions; concerns about the data; concerns about the peer review; concerns about the citations.

According to our result, chryseriol is another main activated compound from LJP, and its target proteins include MAPK4, NOS2, PTGS2, and so on. The MAPK signaling pathway has been recognized to be engaged in osteomyelitis and can regulate differentiation, cell growth, and various types of inflammatory reactions [37]. Wu et al. found that MC3T3-E1 cell *S. aureus* infection enhanced TLR2 expression and triggered both JNK MAPK and ERK signaling pathways [38]. *S. aureus* is a major bone infection triggering pathogen that could generate a sizable quantity of powerful pathogenic ingredients, staphylococcal protein A (SPA). Wang et al. found that c-FOS and NFATc1 expression was upregulated by SPA via MAPK signaling activation to promote osteoclastogenesis [37]. So, we hypothesize that a therapeutic effect on COM may be played by chryseriol through MAPK signaling regulation. Nitric oxide (NO) has critical bone cell function effects and is formed via the arginine metabolism by nitric oxide synthase (NOS). The endothelial isoform of NOS (eNOS or NOS3) is fundamentally expressed at small levels in the bone, while inducible NOS (iNOS or NOS2) expression by bone cells is in reaction to inflammatory stimuli. Proinflammatory cytokines including TNF-*α* and IL-1*β* result in NOS2-pathway activation, and pathway-derived NO promotes cytokines and inflammation-induced bone loss [39]. However, Asensi et al. did not observe osteoblasts NOS2 expression by immune histochemistry in all analyzed bone biopsies and indicated there was an association between osteomyelitis development risk and NOS3 polymorphism [39, 40].

## 5. Conclusions

In summary, LJP targets and active compounds in COM treatment were identified in our study. Luteolin, chryseriol, and other chief active components may perform therapeutic properties through IL-6, IL-10, MMP9, VEGFA, AKT1, EGFR, MAKP, and so on targets regulation. Additional research needs to be accomplished to clarify LJP active compounds' specific therapeutic mechanisms. These works may have a great help for precise treatment and efficient drug selection in COM.

## Figures and Tables

**Figure 1:** Construction of the drug-active compounds-target protein-diseases network. (a) Venn plot of the overlapped genes between targets of LJP active compounds and COM-related genes. (b) The network of drug-active compounds-target protein-diseases. The yellow color indicates 45 overlapped genes between target proteins and COM-related genes, and the red color indicates 15 main active compounds.

**Figure 2:** Identification of the hub genes in the drug-active compounds-target protein-diseases network. (a) PPI network of the 45 overlapped genes between targets of the active components of LJP and COM-related genes. (b) Connection degree statistical of the hub genes from overlapped genes.

**Figure 3:** GO function and KEGG enrichment analysis of the target proteins. (a) GO function analysis of the overlapped genes, including BP, CC, and MF terms. (b) KEGG pathway enrichment evaluation of the overlapped genes.

**Table 1:** The active ingredients with antiosteomyelitis from LJP.

Mol ID	Molecule name	OB (%)	DL	Structure
MOL003062	4,5′-Retro-beta,beta-carotene-3,3′-dione, 4′,5′-didehydro-	31.22	0.55	
MOL003044	Chryseriol	35.85	0.27	
MOL000006	Luteolin	36.16	0.25	
MOL000358	Beta-sitosterol	36.91	0.75	
MOL002773	Beta-carotene	37.18	0.58	
MOL002914	Eriodyctiol (flavanone)	41.35	0.24	
MOL000422	Kaempferol	41.88	0.24	
MOL001494	Mandenol	42	0.19	
MOL003124	Xylostosidine	43.17	0.64	
MOL002707	Phytofluene	43.18	0.5	
MOL003036	ZINC03978781	43.83	0.76	
MOL000449	Stigmasterol	43.83	0.76	
MOL001495	Ethyl linolenate	46.1	0.2	
MOL003101	7-Epi-vogeloside	46.13	0.58	
MOL000098	Quercetin	46.43	0.28	
MOL003059	Kryptoxanthin	47.25	0.57	
MOL003128	Dinethylsecologanoside	48.46	0.48	
MOL003095	5-Hydroxy-7-methoxy-2-(3,4,5-trimethoxyphenyl)chromone	51.96	0.41	
MOL003014	Secologanic dibutylacetal_qt	53.65	0.29	
MOL003108	Caeruloside C	55.64	0.73	
MOL003111	Centauroside_qt	55.79	0.5	
MOL003117	Ioniceracetalides B_qt	61.19	0.19	
MOL003006	(-)-(3R,8S,9R,9aS,10aS)-9-Ethenyl-8-(beta-D-glucopyranosyloxy)-2,3,9,9a,10,10a-hexahydro-5-oxo-5H,8H-pyrano[4,3-d]oxazolo[3,2-a]pyridine-3-carboxylic acid_qt	87.47	0.23	

The article "Network Pharmacology-Based Analysis on Lonicera japonica for Chronic Osteomyelitis Treatment" was retracted in 2023. Reasons: unreliable results or conclusions; concerns about the data; concerns about the peer review; concerns about the citations.

**Table 2:** The main activate compounds from *Lonicera japonica* and their target proteins.

Mol ID	Mol name	Target	Symbol
MOL003044	Chryseriol	Nitric oxide synthase, inducible	NOS2
MOL003044	Chryseriol	Prostaglandin G/H synthase 2	PTGS2
MOL003044	Chryseriol	Mitogen-activated protein kinase 14	MAPK4
MOL000006	Luteolin	Prostaglandin G/H synthase 2	PTGS2
MOL000006	Luteolin	Epidermal growth factor receptor	EGFR
MOL000006	Luteolin	RAC-alpha serine/threonine-protein kinase	AKT1
MOL000006	Luteolin	Vascular endothelial growth factor A	VEGFA
MOL000006	Luteolin	Matrix metalloproteinase-9	MMP9
MOL000006	Luteolin	Interleukin-10	IL-10
MOL000006	Luteolin	Interleukin-6	IL-6

**Table 3:** Chronic osteomyelitis-related genes.

Symbol	Description	Category	Gifts	GC ID	Relevance score
TNF	Tumor necrosis factor	Protein coding	53	GC06P033397	78.55
IL-1RN	Interleukin 1 receptor antagonist	Protein coding	50	GC02P114906	74.66
IL-6	Interleukin 6	Protein coding	51	GC07P022765	72.88
IL-1B	Interleukin 1 beta	Protein coding	50	GC02M112829	64.29
IL-10	Interleukin 10	Protein coding	49	GC01M206767	59.23
IFNG	Interferon gamma	Protein coding	50	GC12M068064	54.49
NLRP3	NLR family pyrin domain containing 3	Protein coding	48	GC01P247415	49.32
CYBB	Cytochrome B-245 beta chain	Protein coding	48	GC0XP037780	49.18
TERT	Telomerase reverse transcriptase	Protein coding	53	GC05M001253	46.16
TNFSF11	TNF superfamily member 11	Protein coding	49	GC13P042562	45.89

## Data Availability

The data used to support the findings of this study are included within the article and are available from the corresponding author upon request.

## Abbreviations

AGE: Advanced glycation end products
AKT1: Protein kinase B
ALB: Albumin
BP: Biological process
CC: Cellular components
CCL2: C-C chemokine ligand 2
CXCL2: Cysteine-X-cysteine motif ligand 2
CXCL8: Cysteine-X-cysteine motif ligand 8
CXCL10: Cysteine-X-cysteine motif ligand 10
CYBB: Cytochrome B-245 beta chain
DL: Drug-likeness
EGFR: Epidermal growth factor receptor
FDR: False discovery rate
ERK: Extracellular signal-regulated kinase
eNOS: Endothelial isoform of NOS
GO: Gene ontology
ICAM1: Intercellular adhesion molecule-1
IFNG: Interferon gamma
IL-1*α*: Interleukin1alpha
IL-1*β*: Interleukin1beta
IL-1RN: Interleukin 1 receptor antagonist
IL-6: Interleukin 6
IL-10: Interleukin 10
JNK: c-Jun-N-terminal kinase
KEGG: Kyoto Encyclopedia of Genes and Genomes
MAPK14: Mitogen-activated protein kinase 14
MF: Molecular functions
MMP1: Matrix metallopeptidase 1
MMP9: Matrix metallopeptidase 9
NFATc1: Nuclear factor of activated T cells c1
NLRP3: Nod-like receptor family pyrin domain containing 3
NOS: Nitric oxide synthase
NOS2: Nitric oxide synthase 2
NOS3: Nitric oxide synthase 3
NO: Nitric oxide
iNOS: Inducible NOS
OB: Oral bioavailability
PPI: Protein-protein interaction
PTGS2: Prostaglandin endoperoxide synthase 2
RAGE: Receptor for advanced glycation end products
SPA: Staphylococcal protein A
TCMSP: Traditional Chinese Medicine Systems Pharmacology Database and Analysis Platform
TERT: Telomerase reverse transcriptase
TLR2: Toll-like receptor 2
TNF: Tumor necrosis factors
TNFSF11: TNF superfamily member 11
TNF-*α*: Tumor necrosis factors-alpha
VEGFA: Vascular endothelial growth factor A
VEGF: Vascular endothelial growth factor.

The article "Network Pharmacology-Based Analysis on Lonicera japonica for Chronic Osteomyelitis Treatment" was retracted in 2023. Reasons: unreliable results or conclusions; concerns about the data; concerns about the peer review; concerns about the citations.

## Supplementary Materials

Supplementary Materials Supplementary Table 1: target symbol, 204 target proteins. Supplementary Table 2: GeneCards search results 686 COM-related genes from the GeneCards database.
